The article "Performance Evaluation of SeisTutor Using Cognitive Intelligence‐Based “Kirkpatrick Model”" was retracted in 2023. Reasons: signs of a paper mill; compromised peer review; unreliable results or conclusions.

# Performance Evaluation of SeisTutor Using Cognitive Intelligence‐Based “Kirkpatrick Model”

**DOI:** 10.1155/2022/5092962

**Published:** 2022-04-16

**Authors:** Ninni Singh, Vinit Kumar Gunjan, Ramana Kadiyala, Qin Xin, Thippa Reddy Gadekallu

**Affiliations:** ^1^Department of Computer Science and Engineering, CMR Institute of Technology, Hyderabad, Telangana 501401, India; ^2^Department of Information Technology, Chaitanya Bharathi Institute of Technology, Hyderabad, Telangana, India; ^3^University of the Faroe Islands, Faroe Islands, Denmark; ^4^Department of Information Technology, Vellore Institute of Technology, Vellore, Tamilnadu, India

## Abstract

The classroom learning environment facilitates human tutors to interact with every learner and get the opportunity to understand the learner's psychology and then provide learning material (access learner prior knowledge and well align the learning material as per learner requirement) to them accordingly. Implementing this cognitive intelligence in intelligent tutoring system is quite tricky. This research has focused on mimicking human tutor cognitive intelligence in the computer-aided system of offering an exclusive curriculum to the learners. The prime focus of this research article is to evaluate the proposed SeisTutor using Kirkpatrick's four-phase evaluation model. Experimental results depicting the enhanced learning gain through intelligence incorporated SeisTutor as against the intelligence absence are demonstrated.

## 1. Introduction

Understanding “Seismic Interpretation” has been considered as important and valuable for petroleum exploration because it provides a sophisticated way of delineating the Earth's subsurface (in the form of seismic snap), understanding the seismic snaps, and then concluding the presence of hydrocarbon or not. This technique can be applied again and again while capturing, analyzing, interpreting, and predicting the presence of hydrocarbon amassing [1].

The interpretation of seismic snaps is a challenging task for a seismologist. Seismologists utilize their expertise to interpret seismic images. However, one possibility is that different geologists interpret the same seismic snap differently during interpretation. This vagueness is due to a lack of thumb rules—the interpretation expertise gained by experience over past years. Thus, novice geologists in this field took many years to gain these expertises. It will be paramount for them if these skills are offered to them at the beginning of their interpretation career. To accomplish this, exploratory learning would be the best strategy for learning. In this learning, an individual has control over the learning process. It means the learner chooses his/her topics, level of difficulty, learning pace, and so forth [2]. To effectively meet this learner-centric requirement, an intelligent tutoring system can offer personalized learning experiences to learners. Intelligent tutoring system (ITS) is an artificial intelligence (AI) technique that provides the learner exclusive learning material, aligned and gathered as per learner grasping ability and preferred media of learning.

SeisTutor has been developed for learning “Seismic Data Interpretation” as a subject domain of this research. This research aims to provide pastoral care to learners by cost-effectively offering one-to-one, customized learning material. SeisTutor delivers a personalized learning environment. It brings personalization in identifying tutoring strategy (based on pretest (learning style test and domain knowledge test)), exclusive curriculum design, and observation of learner psychological state of mind during learning sessions. The feature of personalization is built on many aspects, such as accuracy of predicting tutoring strategy (based on pretest), curriculum design, and psychological parameters. The only technique to determine the performance of the personalization facility of SeisTutor is to appraise the system in actual circumstances (learners who are learning the course material). Appraise acts as a critical element for quality assurance because it enables the learner to give their valuable feedback on learning experience and on learning content, which further helps to understand the learner perspective and makes the learning better.

The evaluation of SeisTutor was accompanied in the 2018–2019 academic year. The objective of the assessment is to examine how effectively SeisTutor personalized itself to fulfill the learner's needs and whether SeisTutor helps enhance the learning gain for learning the “Seismic Data Interpretation” domain. To accomplish this, the following program is outlined:

1. Perform schematic literature review on how to evaluate the efficacy of learning.
2. Generate an assessment for determining the effectiveness of learning.
3. Perform analysis to identify how efficiently learners learn with SeisTutor.

This article is organized into five sections. It begins with a schematic literature review on evaluation on learning with ITS (Section 2). Further, Section 3 introduces the architecture of SeisTutor in detail, which includes the general description and mathematical justification of its functionalities.  Section 4 illustrates the experimental analysis performed to evaluate the effectiveness of SeisTutor systematically.  Section 5 elaborates the comparative analysis with current work, and, in Section 6, we finally conclude the paper with the implication of this work.

## 2. Background and Preliminaries

Evaluating and validating an ITS is a challenging task due to the lack of standard agreement and procedure.

The primarily used prototype for evaluating the training program of ITS is the prototype established by Donald Kirkpatrick [3–6]. Many researchers have revised this prototype, but its basic architecture is still the same [7].

Kirkpatrick's prototype comprises four stages of evaluation shown in Figure 1 and briefly discussed in Figure 2.

Computing results is the best way to quantify the effectiveness of any learning program, but it is challenging to conduct. McEvoy and Buller [13] put a statement regarding evaluation that not all learning programs focus on impacting the learning performance of a learner; instead, they can perform for a purpose. Other researchers used the Kirkpatrick model as a base model. Philips [14] introduced the fifth level on Kirkpatrick model named Return of Investment (ROI), used to measure the effectiveness of learning or investment.

The authors in [15] considered Kirkpatrick's model as a base model for measuring the effectiveness of a learning program. Their suggestion is to set the initial objective (from the learning program) and then monitor the fulfillment of objectives after the learning program. References [16, 17] disapproved Kirkpatrick's model by giving the following reason:

- Offline Test (Written Test) lacks validity and reliability in quantifying knowledge, skill, and attitude (KSA).
- 100% response rate is idealistic.
- Control groups are not feasible in the learning program context.

Furthermore, educational organizations have recommended considering the merits and demerits of various evaluation prototypes and methodologies to build an organizational-specific evaluation prototype that fulfills their requirements [18]. In addition to this, it has been suggested that the evaluation prototype emphasizes both education processes and their outcomes [19]. Valid, reliable, inexpensive, and acceptable are the features of an ideal evaluation prototype. Moreover, the evaluation prototype may encompass quantitative, objective, subjective, and qualitative methods. Thus, evaluation results are advantageous for determining the learning attainments of the learning program [17, 20, 21].

The conclusion drawn from the literature recommends that the learning program include three levels of Kirkpatrick's prototype. Kirkpatrick level 3 and level 4 are very challenging to observe in an educational learning program [22] because while level 1 and level 2 can be quantified during an ongoing learning session, level 3 and level 4 require postassessment analysis. Level 4 needs the rigorous observation of the inference of the learning program. For evaluation, there is no articulated framework. As per [23], continuous feedback and instruction help the learner to achieve best in learning skills Storch and Tapper [24]; Polio et al. [25] Elliot and Klobucar [26]; Aryadoust et al. [27].

## 3. SeisTutor Functionality

This section illustrates the SeisTutor architecture and briefly discusses functionality incorporated in SeisTutor. SeisTutor is an ITS explicitly designed for the “Seismic Data Interpretation” subject domain. SeisTutor recommends learning contents as per learner performance in pretest (prior knowledge assessment test). In addition, SeisTutor keeps track of the learner's behavior (psychological state) during the entire learning session and conducts a test to determine the degree of understanding of the topic. SeisTutor is adaptive, that is, content and link-level. Adaptive content level indicates that the learners with different performance in pretest (prior knowledge test) get different learning material. Before indulging learners in the learning session, SeisTutor enables learners to go through a pretest. There are two kinds of assessments performed in pretest: a learning style test and a prior knowledge test. The current focus of this research is on the prior knowledge test. SeisTutor observes the learner's performance during the tests and aligns the learning material accordingly.

For link elimination, ideally, the curriculum covers all the links of subtopics to learn; however, the links eliminated are not in the determined curriculum for the learner. SeisTutor continually observes and stores the learner's action, performance, and behavior. This information is further utilized for making intelligent strategic plans for recommendation and evaluation work.

## 4. SeisTutor Architecture

SeisTutor follows all the guidelines for implementing an intelligent tutoring system. The critical functional model of an ITS is the domain model, learner model, pedagogy model, and learner interface. SeisTutor architecture comprises learner model, pedagogy model, domain model, and learner interface (architecture paper). The following subsection briefly illustrates the various components involved in SeisTutor.

### 4.1. Domain Model

The domain model is described as the cluster of concepts. Here concept terminologies indicate the single topic. Other terminologies are used in the different research papers, such as knowledge element, object, learning outcome, and attribute. In the current context, concepts possess a prerequisite relationship to each other. Each concept is further segregated into learning units. SeisTutor utilizes unit variant technologies to attain content-level adaptation. Content-level adaptation indicates that the system has alternative units and recommends the learning units based on learner grasping and learning style.

### 4.2. Pedagogy Model

The pedagogical model consists of various rules and logic that build a knowledge infrastructure essential for adapting the learning materials as per the learner's.

 
*Curriculum planner*: The planner generates a curriculum as a sequence of learning units to be covered during the learning session [28].
 
*Learning assessment*: Learning assessment is the process of determining the learner's learning process. The accuracy of this adjudging model acts as a critical factor that affects the adaptation practice.
 
*Understanding assessment*: Understanding assessment identifies the learner's degree of understanding of the concept. SeisTutor makes any decision by referring to all the models like determining the curriculum for the learner and offering the learning content as per learner grasping level and learning style.

### 4.3. Learner Model

The learner model captures the learner's activity during the learning session and stores and updates the learner's information for making the decision. This information is fruitful for the system to adapt based on learner characteristics (grasping level and learning style). SeisTutor captures three characteristics of a learner.

 
*Learner demographic information*: Learner demographic information includes learner's basic details, such as name, learner username, and e-mail id. This information is used to create the learner profile and collected when the first-time learner signs up with SeisTutor.
 
*Psychological state*: It recognizes the learner's emotions during the tutoring session. Recognizing the psychological state of mind is essential because it helps determine how far the learner liked the learning contents during the learning session. SeisTutor determines six emotions, that is, happy, sad, neutral, surprised, afraid, and angry.

This **psychological state** recognition module gets triggered as soon as the learner starts the learning session, as shown in Figure 3. Initially, participants belong to both studies and undergo the initial assessment phase (pretest); after pretest, their learner profile and learning style are determined. The I2A2 learning style prototype is utilized to ascertain the learning style. Based on the tutoring strategy (study 2 and study 1) and course coverage plan, the learner and pedagogy model determine the relevant learning mode (study 1) and represent the learning contents delivered using the learner interface. Thus, SeisTutor examines the participant's attainment in pretest and predicts the individualized tutoring strategy (study 2 and study 1) and custom-tailored curriculum for the applicants (study 1).

As illustrated in Figure 4, the CNN-based emotion recognition module is instantiated as soon as the learner begins the learning session. This emotion recognition module takes the snap of the learner via webcam, which acts as an input to the CNN-based emotion recognition module. This module determines the learner's psychological (emotion) state, which is gauged for future analysis (phase 1: evaluation of reaction). The gathering psychological (emotion) state is repeated until the learner completes all the learning contents (topics) associated with all the weeks.

### 4.4. Min-Max Normalization

The learner classification parameters (prior knowledge test (0–5), postassessment test (0–5), learning gain (0–5), and learner emotion (0–100)) of each learner were used and normalized using the method called Min-Max. It converts a value of *Y*={*y*_1_, *y*_2_, *y*_3_,…, *y*_*n*_} and converges in the range of [*A*, *B*]. The formula for score standardization is specified below, where *A* is the lowest range and *B* is the highest range. In our case [*A*, *B*] is [0, 10];

(1) $$\begin{array}{c} Z=\left\{\frac{y_{i}-\text{Lowestvaluein}Y}{\text{Highestvaluein}Y-\text{Lowestvaluein}Y}\right\}*\left(B-A\right)+A. \end{array}$$

**Learner performance** evaluates the learner's performance by quantifying the learner's learning by organizing quizzes and tests.

### 4.5. Quiz and Understanding Test Representation

Learner performance has been quantified based on one parameter, that is, the number of correct responses. As soon as the learner finishes the learning content of each week, he or she has to give a quiz and understanding test. One quiz is associated with every week (shown in Figure 5). Each quiz contains five questions, and each question contains only one hint. Hints appear to the learner based on the learner's request to seek help to solve the question. SeisTutor asks the learner to summarize the learned concepts in understanding the test. Based on the user entered information, dictionary-based sentimental analysis is performed. The result gives a score out of 100, which tells the learner's overall understanding of the concepts.

To determine the overall learning gain, SeisTutor has pretest and posttest assessment scores. The average learning gain is computed (using the following equation):

(2) $$\begin{array}{c} \text{Learning}\_\text{Gain}=\;\left({\text{PostTest\_Score}}_{\text{L}}{-\text{PreTest\_Score}}_{\text{L}}\right). \end{array}$$

#### 4.5.1. Learning History

It keeps track of the learner's activity, such as login time and total time spent, and its interaction details during the entire tutoring sessions.

SeisTutor utilizes this information to make necessary action which further helps to make the whole learning process effective.

To start tutoring with SeisTutor, the learner needs to register himself/herself first (see Figure 6). After registration, SeisTutor creates a learner account and instructs the learner to give a pretest. Pretest comprises two tests:

1. Prior knowledge test
2. Learning style test

### 4.6. Prior Knowledge Test

The prior knowledge test is the preliminary test used to identify the domain's elementary knowledge to know the learner's initial learning level. This test is responsible for analyzing the learner's knowledge about the domain. The domain model examined the test result and categorized the learners into three learning profiles, that is, “beginner, intermediate, and expert” (see Figure 7). A further outcome of this result is also responsible for determining the curriculum, which is exclusively designed for the learner. This test comprises twenty questions, and all the questions are verified by the domain expert of Seismic Data Interpretation.

### 4.7. Learning Style Test

This test is responsible for determining preferred media for learning. The research has noticed that learner performance is gradually increased if learning material is provided as per preferred learning media (see Figure 3). Thus, this test analyzes the learner-preferred media. The learner model examines the test result and categorizes the learners into four learning styles, that is, “Imagistic, Acoustic, Intuitive, and Active.”

Based on these two tests, the pedagogy model determines the tutoring strategy (the result of learning profile and learning style). A tutoring session then begins with the determined tutoring strategy. As soon as learning begins, psychological features get triggered, capturing learner emotions and saving the results in the database for future reference. After completion of every week, the learner is tested. Based on the test result, learner performance and degree of understanding are computed.

## 5. Results and Discussions

After tutoring, posttutoring assessments of learners are performed by SeisTutor (see Figure 8). This section depicts the analysis used to determine the impact of study 2's learning methods with SeisTutor. It exercises learning practices with features like personalized curriculum design and recognition of the psychological state of the learner during the learning process, and learner's degree of understanding of taught concepts is characterized as study 2. When it is not practiced, it is characterized as study 1. An experimental comparison of both study groups is tabulated (Table 1). These variances help to identify the discrepancy in the learning experiences.

### 5.1. Experimental Design and Methodology

The SeisTutor evaluation is the fundamental piece of the development of this framework. In order to quantify the adequacy and effectiveness of SeisTutor, assessment tests have been conducted. SeisTutor has been tested on a selected population of students, teachers, and both (teachers and students) from an anonymous university. A total of 60 learners volunteered in the evaluation process. Based on their compliance in the participation, a compliance agreement form was issued which demonstrates essential details related to the assessment process. It is a requisite for each applicant to give their approval for participation in the assessment process. Applicants were haphazardly assigned one of the groups. 32 applicants were in study 1, and the remaining were in study 2.

Out of 60 learners, 30% are learners pursuing graduation, 17% are graduates, 35% are postgraduates, and the rest's minimum qualification is doctorate (Ph.D.).

12% of learners were in the 18–20 age group, 18% of learners were in the 20–22 and 22–24 age groups, 5% of learners were in the 24–28 age group, 12% of learners were in the 28–32 age group, 22% of learners were in the 32–34, and the rest were in the above 34 age group (shown in Table 2). SeisTutor is explicitly created for the “Seismic Data Interpretation” domain. As a result, it is intended to be used by participants or learners belonging to the petroleum engineering and exploration domain. Thus, to quantify the effectiveness of SeisTutor, undergraduate learner (B.Tech/B.E. Petroleum Engineering), teacher (Petroleum Engineering Dept.), and others (government exploration industry) are taken into consideration (see Table 2).

The learners underwent a pretest as soon as they got registered with SeisTutor. Their learning style and grasping level (learning level) were adjudged as 28 learners as mentioned above were in study 2. Based on their responses in the pretest, the custom-tailored curriculum is determined, which is realigned and reorganized from the domain (content) capsule. SeisTutor examines every learner involved in study 2, identifies their psychological state (emotions) during the learning session, and quantifies the degree of understanding about the concepts. The remaining learners in study 1 follow the standard curriculum for learning, that is, contents in the same sequence (irrespective of their prior knowledge about the domain). Thus, all the learners follow the same learning path. The point to underline is that their pretest performance is not used for exclusive learning path recommendations. The learning session begins week-wise for both the study groups and subsequent postassessment tests.

### 5.2. Data Preparation

Before analysis, obtained data underwent data screening phase. In this phase, the elimination of missing values and data normalization is performed. For deducing conclusion about the effectiveness of learning through SeisTutor, learner's performances, that is, prior knowledge test (pretest), understanding test, psychological state results, and quiz test (posttest) during learning, are taken into consideration. SPSS version 25 was used for accomplished analysis.

### 5.3. Result Discussion

The evaluation of SeisTutor is performed using the Kirkpatrick evaluation model. As discussed in Section 2, the Kirkpatrick evaluation prototype comprises four phases shown in Figures 1 and 2.  Table 3 describes the statistical methods and performance metrics used in the four levels of evaluation.

### 5.4. Kirkpatrick Phase 1: Evaluation of Reaction

Evaluation of reaction as its name indicates is the evaluation of the reaction (emotion) of the learner during learning or how far the learner likes the learning content and teaching process, that is, pedagogy. SeisTutor incorporates an emotion recognition module and an open-end questionnaire (learner feedback).

The Min-Max normalization is utilized to maintain the uniformity, which converges the original values in the scope of [0–10].

As mentioned in Table 1, the psychological state of the learner is determined only for the applicants involved in study 1. Thus, their descriptive states are shown in Table 4. From the stats shown in Table 4, the average mean score percentage among 28 applicants is 44% for emotion happy, 40% for emotion neutral, 36% for emotion angry, 32% for emotion surprised, 30% for emotion afraid, and 24% for emotion sad. Thus, one can deduce with confidence that, on average, learners are happy with the learning content and teaching process, that is, pedagogy.

### 5.5. Kirkpatrick Phase 2: Evaluation of Learning

Evaluation of learning, as its name indicates, is the evaluation of how effectively learners grasp the learning content. SeisTutor conducts a small quiz and degree of the understanding test to adjudge the learner's overall learning.

The average learning gain of applicants involved in study 1 is 22% and in study 2 it is 12%. Thus, it is concluded that if learning material is offered as per the learner's inclination with an exclusively designed curriculum based on the learner's prior knowledge, then the proposed SeisTutor succeeds in enhancing the learner curiosity and interest, which indirectly enhances the overall learning gain (see Table 5 and Figure 9).

These tests were performed on learning gain and degree of understanding of study 1 through SeisTutor. Table 4 illustrates the progressive learning gain of 22% discovered among learners, those applicants who participated in study 1 of SeisTutor. Furthermore, this information (statistical) is used in analysis, that is, bivariate Pearson correlation.

Understanding tests were designed and conducted only for study 1 because it strongly proves the effectiveness of learning gain achieved by intelligent feature incorporated SeisTutor. Here, the correlation of learning gain with itself is one because a variable or parameter is perfectly interrelated. The Pearson correlation of learning gain with degree of understanding is 0.484, and the two-tailed significance, that is, *P* value, is less than 0.01 (see Tables 6 and 7). Thus, one can confidently say that learning gain and degree of understanding have statistically significant linear relationships (see Figure 10).

### 5.6. Kirkpatrick Phase 3: Evaluation of Behavior

Evaluation of behavior is quite hard to quantify. To measure this, SeisTutor collects feedback from the applicants. As the learner completes all the learning concepts of every week, SeisTutor requests the learner feedback. In this section, a conclusion from the learner feedback is drawn. Learners who have been the impeccable part of this evaluation of SeisTutor had a good perception of the system, and their feedbacks are very encouraging. It has appeared in their reactions whether they would like to recommend SeisTutor to others who need to take this study. Around 93% of the learners showed that they would recommend it to others, out of which 48% showed strong agreement, and the remaining 45% agreed on a recommendation as well (see Table 7). The overall satisfaction with SeisTutor was around 93%, out of which 45% were strongly satisfied and 48% were satisfied. It has also been observed that learners' studies became productive with SeisTutor (Table 8).

Few questions were asked on the impact of the intelligent features provided by SeisTutor and they are collected and summarized in Table 9. As some intelligent feature is not provided for study 2 applicants, 28 effective feedback from study 1 participants have been taken into consideration.

Most of the participants were happy with the tutoring strategy provided by the system, with 86% satisfaction, which includes 46% who were satisfied and 40% who were strongly satisfied. 85% of participants felt that learning by their own made them perform better, with 40% being strongly satisfied and 45% being satisfied. The participants were happy with the recommended exclusive curriculum by the system with 85% satisfaction, with 35% being satisfied and 50% being strongly satisfied. Most of the participants were happy with the recommended custom-tailored curriculum provided by the system, with 85% satisfaction, with 39% being satisfied and 46% being strongly satisfied. 92% of participants agreed that the understanding test at each week corresponds to the lesson taught; 39% strongly agreed, and 53% agreed. At last, 82% of students agreed with the psychological parameter accurately determined with SeisTutor: 39% strongly agreed to this and 43% agreed.

The overall impact of the support provided by SeisTutor on the learning process is assessed through the learner's feedback questionnaire answered by 60 participants (see Table 10). The analyzed results showed that 87% of the students are happy with SeisTutor supports, with 47% satisfied and 40% strongly satisfied. In addition, 78% of the students are happy with the system navigation support to find the needed information, with 43% satisfied and 35% strongly satisfied. At last, there was 80% satisfaction among the students, out of which 42% had a strong agreement and 38% agreed that the SeisTutor prelearning procedure was beneficial for learning.

The usefulness of the lesson components such as lesson explanations, revisions, presented quizzes, and the question hints in the learning process was evaluated in Table 11. The questionnaire feedback results show that 85% of students were happy with the content explained by SeisTutor, with 47% satisfied and 38% strongly satisfied. Moreover, 78% of students showed interest and agreed that the tutoring resources were adequate, with 35% strongly satisfied and 43% satisfied. It is clear that the quizzes and hints were realistic and focused with the learning contents provided by SeisTutor.

The impact of the interactive graphical user interface, content organization, and design features of SeisTutor in the learning process is evaluated through the learner questionnaire responses, described in Table 12. The questionnaire results revealed that there was 77% satisfaction with the interactive GUI and content organization of SeisTutor among the learners, with 40% strongly satisfied and 37% satisfied. There was 80% satisfaction with SeisTutor to compel and support to complete the quizzes and lessons among the learners, with 44% strongly satisfied and 36% satisfied. Finally, students were happy with the account setup process with the system, which maintains the learners learning progress, grades, and basic account information.

The learner's overall evaluation of the SeisTutor showed that 82% of learners agreed that tutoring should begin based on the learner profile considering his/her learning style and prior knowledge. Most of the students were unaware of their learning style, and about 80% of students never knew about it. Most of the students liked the artificial intelligence features such as automatic selection of the tutoring strategies, dynamically assessing the learner attainment and flipping the tutoring plan or strategy.

The learner's feedback questionnaire responses were retrieved and analyzed in an accessible fashion. Some learners put their suggestions to improve the productivity of SeisTutor. Most of the suggestions were general and related to the improvement of the system, and few were pessimistic regarding improvement of the quality of learning contents, improving the quality of the video lessons, and hints provided by the system. At last, through the overall evaluation of SeisTutor, 87% of learners agreed that they improved their learning performance and outcomes.

### 5.7. Kirkpatrick Phase 4: Evaluation of Results

Evaluation of results illustrates the overall impact of learning on the learner. To quantify the effectiveness of learning, paired-wise sample *t*-test is performed on existing information, that is, pretest and posttest results of participants involved in both studies (study 1 and study 2). Here two cases are taken into consideration.

Case 1: A paired-sample *t*-test accomplished on study 1 incorporates the cognitive intelligence (see Table 1).
    Hypothesis Case 1.0. Let us assume that the applicants involved in study 1 have homogenous mean scores in pretest and posttest.
    Hypothesis Case 1.1. Let us assume that the applicants involved in study 1 did not have homogenous mean scores in pretest and posttest.
Case 2: A paired-sample *t*-test accomplished on study 2 incorporates the cognitive intelligence (see Table 1).
    Hypothesis Case 2.0. Let us assume that the applicants involved in study 2 have homogenous mean scores in pretest and posttest.
    Hypothesis Case 2.1. Let us assume that the applicants involved in study 2 did not have homogenous mean scores in pretest and posttest.

For study 1, the calculated *T* value (*T*_Stats_, *p* < 0.01) is 11.410 (refer to Tables 13 and 14). The difference between posttest and pretest scores is 2.21786, and the calculated *T*_Stats_ value exceeded the *T*_critical_ value. Therefore, Hypothesis 1.0 is excluded. Tables 13 and 14 Indicate a considerable difference between pretest and posttest scores. For study 2, the calculated *T* value (*T*_Stats_, *p* < 0.01) is 5.312 (refer to Tables 15 and 16). The difference between the posttest and pretest scores is 1.24719, and the calculated *T*_Stats_ value exceeded the *T*_critical_ value. Therefore, Hypothesis 2.0 is excluded. Tables 15 and 16 indicate a considerable difference between pretest and posttest scores. Both studies excluded the null hypothesis, implying that both provide useful training. On the other hand, this study determines which study has the most significant influence on improving learning gains. In order to deduce the conclusion, the objectives of both studies are compared. Study 1 achieved high scores compared to study 2. As a result, study 1 differs significantly from study 2 in posttutoring and pretest results, indicating that study 1 provides a more effective training program.

This analysis concludes that the intelligent incorporated SeisTutor used in study 1 outperforms SeisTutor used in study 2 in providing custom-tailored intended curriculum, identifying learner sentiments while learning, and computing the learner's overall degree of knowledge that meets the learner needs.

## 6. Conclusion

This article demonstrates the proposed personalized intelligent tutoring system, named SeisTutor. From the research, it has been noted that a learner receives repetitive learning content from learning, which indirectly disorients the learner. Thus, to address this issue, bug model has been utilized, which analyzes the bugs and recommends the custom-tailored curriculum to the learner. This technique helps to bring empathy to ITS. SeisTutor is not a passive tutor; it also analyzes the learner's behavior, that is, the psychological state of the learner during learning, which helps to understand the learner's experience with SeisTutor (about learning content). Experimental results reveal that SeisTutor utilized by participants in study 1 provides a customized learning sequence or path of learning material that endorses effective learning. Experimental analysis reveals the effective learning gain (when learner gets the custom-tailored sequenced learning material) of 44.34% compared to SeisTutor used in study 2 (not sequenced learning material). To evaluate the overall effectiveness of SeisTutor, Kirkpatrick's four-phase evaluation model is utilized. The analysis reveals that the participants involved in study 1 attain 44.4% while study 2 attains 24.8% and study 1 provides effective learning.

## Figures and Tables

**Figure 1:** Kirkpatrick's four stages of evaluation.

**Figure 2:** Brief illustration of Kirkpatrick's four stages of evaluation [8–12].

**Figure 3:** Flow of learning style test (LST) questionnaire.

**Figure 4:** Flow diagram of CNN-based emotion recognition module.

**Figure 5:** Quiz and understanding test representation.

**Figure 6:** Flow diagram of learner characteristics model.

**Figure 7:** Flow of domain knowledge test (DKT).

**Figure 8:** Flow of accomplishing the evaluation process.

**Figure 9:** Learning gain of study 1 and study 2.

**Figure 10:** Linear relationship with learning gain and degree of understanding.

**Table 1:** Feature of study 1 and study 2 evaluation groups.

	Study 2	Study 1
Personalized tutoring contents	Offer learning content (similar curriculum) based on tutoring strategy	Offer personalized learning content (different curriculum) based on determined prior knowledge level and tutoring strategy [29, 30]
Psychological state tracking	Psychological state of the learner is not tracked during ongoing learning session	Determine psychological state of the learner during ongoing learning session
Degree of understanding computation	Learner's understanding about the concept is not adjudged	Quantify learner's understanding about the concept

**Table 2:** Learner demographic characteristics.

Demographic characteristics			
Characteristic		*N* = 60	
		Frequency	Percentage (%)
Gender	Male	35	58
	Female	25	42

Age	(18–20)	7	12
	(20–22)	11	18
	(22–24)	11	18
	(24–28)	3	5
	(28–32)	7	12
	(32–34)	13	22
	(>34)	8	13

Qualification	Diploma	0	0
	High and secondary school	18	30
	Graduation	10	17
	PG	21	35
	Ph.D.	11	18

Occupation	Student	18	30
	Teacher	11	18
	Both (student and teacher)	19	32
	Others	12	20

**Table 3:** Statistical and performance metrics considered for four-phase evaluation.

Kirkpatrick levels	Statistical methods	Performance metrics
Level 1: evaluation of reaction	Average mean score analysis	Emotion parameter
Level 2: evaluation of learning	Average mean score analysis	Learning gain
	Bivariate Pearson correlation	Degree of understanding

Level 3: evaluation of behavior	Average mean score analysis (learner feedback)	Effectiveness
		Overall satisfaction
		Adaptation & personalization
		Satisfaction level on custom-tailored curriculum sequencing recommendation module

Level 4: evaluation of results	Paired-wise sample *t*-test (hypothesis analysis)	Pretest and posttest scores

**Table 4:** Descriptive statistics of psychological parameter of learner for study 1.

Emotions	Mean (/10)	Std. deviation	Mean (%)
Happy	4.4174	29.6357	44
Sad	2.4272	24.9175	24
Surprised	3.2275	28.2939	32
Afraid	3.0612	26.8571	30
Angry	3.6728	26.1069	36
Neutral	4.0389	26.6193	40

**Table 5:** Learner's learning gain.

Study cases	Number of participants (*n*)	Learning gain		
		Mean (/10)	Standard deviation	Mean (%)
Study 1	28	2.2170	1.02795	22
Study 2	32	1.2793	1.37034	12

**Table 6:** Average mean score of learning gain and degree of understanding.

Study 1 parameters	No. of participants (*n*)	Learning gain		
		Mean (/10)	Standard deviation	Mean (%)
Learning gain	28	2.2170	1.02795	22
Degree of understanding	28	2.5467	1.31201	25

**Table 7:** Correlation matrix between learning gain and degree of understanding.

Parameters		Learning gain	Degree of understandings
Learning gain	Pearson correlation	1	0.484^*∗∗*^
	Sig. (2-tailed)		0.009
	N	28	28

Degree of understanding	Pearson correlation	0.484^*∗∗*^	1
	Sig. (2-tailed)	.009	
	N	28	28

^*∗∗*^Correlation is significant at the 0.01 level (2-tailed).

**Table 8:** Learner feedback on effectiveness of SeisTutor.

	Questions	Degree				
		Strongly satisfied	Satisfied	Neutral	Dissatisfied	Strongly dissatisfied
System effectiveness	What is your overall level of satisfaction with SeisTutor?	27	23	6	3	1
	The learning through this tutoring system (SeisTutor) was easy	27	26	5	1	1
	Did you feel that you were achieving learning outcomes?	30	21	6	3	0
	I would recommend a course through SeisTutor with no instructor help	29	24	3	5	0
	Would you recommend SeisTutor to individual who needs to take another course?	25	27	5	3	0
	Did SeisTutor support you to make your study productive?	28	27	3	0	2
	How well does this system deliver on your learning intentions?	31	21	5	2	1

**Table 9:** Learner feedback on adaptivity of SeisTutor.

	Questions	Degree				
		Strongly satisfied	Satisfied	Neutral	Dissatisfied	Strongly dissatisfied
Adaptivity/personalization	Did SeisTutor satisfy you with dynamic creation of your learning profile?	27	21	7	1	4
	Were you convenient and satisfied with the tutoring strategy presented to you by SeisTutor?	24	19	9	6	2
	The information provided by SeisTutor is at a level that you understand	29	17	12	0	2
	The tutoring session was at the right level of difficulty for me	26	23	9	2	0
	As a learner, did you feel that your learning style was appropriately judged?	29	25	3	2	1
	Once tutoring begins and you were tutored, were your learning preferences sufficiently satisfied?	24	24	9	2	1
	Did the experience of learning by your own learning preference make you perform better?	24	21	6	7	2
	Based on your prior subject knowledge, has SeisTutor accurately determined exclusive curriculum for you?	14	8	2	3	1
	How satisfied are you with the exclusively determined curriculum?	13	7	4	3	1
	As a learner did you feel learning material enabled you to improve your ability to formulate and analyze the problem?	10	14	1	3	0
	Are you satisfied with the sequencing of learning content?	14	09	3	2	0
	Does sequencing of learning material relate with your prior knowledge? (give rating)	12	11	2	3	0
	Does learning content formulated under various learning levels and styles satisfactorily justify itself? (give rating)	17	7	2	0	2
	Has this learning session been successful in improving your knowledge in the subject domain? (give rating)	12	11	2	3	0
	Did this learning material fulfill your expectations?	11	13	2	1	1
	The understanding test at the end of each week corresponds to the lessons taught?	11	13	2	0	2
	SeisTutor compels and supports me to complete the quizzes, understanding test, and lessons ?	13	12	2	0	1
	The posttutoring evaluation system (week-wise understanding) as it exists is	14	10	1	2	1
	How do you rate the sequence of the lessons in the course?	18	8	0	0	2
	Has SeisTutor accurately determined your psychological (emotional) state during tutoring session? (give rating)	11	7	5	5	0
	Do you feel recognition of emotion during ongoing tutoring is indicative of empathy of the system?	13	12	2	0	1
	The course contents are relevant and well organized?	14	10	1	2	1

**Table 10:** Learner feedbacks on SeisTutor ongoing learning support.

Questions	Degree				
	Strongly satisfied	Satisfied	Neutral	Dissatisfied	Strongly dissatisfied
How are you satisfied with the system support?	24	17	11	6	2
The system navigation support enabled finding the needed information easily	21	17	9	11	2
Was the prelearning procedure available in SeisTutor helpful to you?	25	17	6	9	3
Were you able to understand the language used to explain the lessons in SeisTutor?	33	21	6	0	0
The tutoring was flexible to meet my learning requirements	30	21	7	2	0

**Table 11:** Learner feedback on learning material, quizzes, and overall SeisTutor support.

	Strongly satisfied	Satisfied	Neutral	Dissatisfied	Strongly dissatisfied
SeisTutor explained the content correctly	23	25	3	8	1
SeisTutor made the course as interesting as possible	31	19	9	1	0
The tutoring resources were adequate	21	19	7	9	4
The presentation of course content stimulated my interest during learning session	32	24	2	1	1
The course contents are relevant and well organized	29	25	3	2	1
SeisTutor supported me to understand the content which was found confusing?	27	26	6	1	0
Did the quiz at the end of each week correspond to the lessons taught?	28	27	3	1	1
The question-wise hints were helpful	27	26	6	0	1
Did the SeisTutor react decidedly to your necessities?	26	21	11	1	1
Was the learning provided sufficiently to take the quiz?	36	18	4	2	0
During ongoing tutoring, assessments are a fair test of my knowledge and learning preferences	32	21	5	2	0

**Table 12:** Learner feedback on learning material presentation and on overall SeisTutor look and feel.

Questions	Strongly satisfied	Satisfied	Neutral	Dissatisfied	Strongly dissatisfied
How satisfied are you with the look and feel (user interface design) of this system?	32	19	8	1	0
How satisfied are you with the account setup experience of this system?	31	21	5	3	0
How pleasing is the color scheme used in this system?	28	21	11	0	0
How user-friendly is this system? give a rating	27	21	8	2	2
SeisTutor compels and supports me to complete the quizzes and lessons	25	27	6	1	1
How satisfied are you with the organization/customization of contents feature of the system?	29	26	4	0	1

**Table 13:** Statistical results of paired-sample *t*-test of study 1.

Comparison item	Learning mode			
	Mean	*N*	Std. deviation	Std. error of the mean
Posttest of study 1 applicants	3.9375	28	.39455	.07456
Pretest of study 1 applicants	1.7196	28	.99740	.18849

**Table 14:** Paired-sampled *t*-test results of study 1.

	Mean	Std. deviation	Std. error of the mean	95% confidence interval of the difference			*T*	d*f*	Sig. (2-tailed)
				Lower		Upper			
Pair 1: posttest of study 1–pretest of study 1	2.21786	1.02856	.19438	1.81902	2.61669		11.410	27	.000

**Table 15:** Statistical results of paired-sample *t*-test of study 2.

Comparison item	Learning mode			
	Mean	*N*	Std. deviation	Std. error + Mean
Posttest of study 2 applicants	3.6525	32	0.58915	0.10415
Pretest of study 2 applicants	2.4053	32	1.39565	0.24672

**Table 16:** Paired-sampled t-test results of study 2.

	Mean	Std. deviation	Std. error of the mean	95% confidence interval of the difference			*T*	d*f*	Sig. (2-tailed)
				Lower		Upper			
Pair 1: posttest of study 2–pretest of study 2	1.24719	1.32804	.23477	.76838	1.72600		5.312	31	.041

## Data Availability

The data used to support the findings of this study are available from the corresponding author upon request (thippareddy.g@vit.ac.in).
